The article "Research on the Training Strategy of Aerobic Physical Education Talents under the Background of Artificial Intelligence Era" was retracted in 2023. Reasons: signs of a paper mill; suspected computer-generated content; unreliable results or conclusions; lack of ethics approval or compliance.

# Research on the Training Strategy of Aerobic Physical Education Talents under the Background of Artificial Intelligence Era

**DOI:** 10.1155/2022/1102760

**Published:** 2022-02-03

**Authors:** Xiaojing Liu, Hong Wang

**Affiliations:** Beijing Sport University, Beijing, China

## Abstract

Aerobic is loved by the public, especially the young people, through the combination of the art and power of dance. With people's attention to health, the demand for aerobic professionals is increasing. As an important training base for aerobic professionals, the level and teaching ability of aerobic professionals have a great influence on students. The gradual maturity and rapid popularization of artificial intelligence bring many opportunities and challenges to the teaching of physical education in colleges and universities. Only by seizing the opportunities and facing the challenges, excavating their own existing problems, and transforming with the help of artificial intelligence can we adapt to the development trend of educational modernization in China. In order to increase the standardization and standardization of aerobics and provide executable standards for aerobic learning, performance, and adjudication, through the research on the training strategy of aerobic sports talents under the background of artificial intelligence era, capture aerobic performance actions with artificial intelligence awareness, standardize and standardize aerobics, and discuss the teaching effect of school intelligent aerobics, it is found that this study not only has important physical education teaching value but also relates to the application prospect of artificial intelligence technology in aerobic physical education talent training strategy.

## 1. Instruction

Aerobics originated from the traditional aerobic exercise, which is a kind of aerobic exercise. It has high requirements for limb coordination and consistency, strength, and movement standard [1]. Aerobic sports refers to a comprehensive sports activity integrating gymnastics, dance, and martial arts with the accompaniment of music. It is a perfect combination of action and music. It has the characteristics of spanning the four fields of sports, education, literature, and medicine. It is also an emerging sports project to cultivate human health and beauty on the basis of ordinary sports [2]. According to the purpose of aerobic teaching activities and the tasks to be solved, it is divided into aerobic performance course, referee course, and teaching course. Aerobic education not only shows the “health” and “strength” of movements but also emphasizes the sense of “beauty.” It perfectly integrates the art of human language and sports aesthetics, makes aerobics a highly ornamental physical education sport, has important physical education value, and is also an important means to promote the physical and mental health of college students [3].

The article "Research on the Training Strategy of Aerobic Physical Education Talents under the Background of Artificial Intelligence Era" was retracted in 2023. Reasons: signs of a paper mill; suspected computer-generated content; unreliable results or conclusions; lack of ethics approval or compliance.

In recent years, due to the rapid development of artificial intelligence technology in the global field, countries all over the world have actively carried out application and research. Some developed countries continue to strengthen the strategic layout and innovation of artificial intelligence technology to enhance national competitiveness [4]. The State Council of China fully deployed the development plan of artificial intelligence in 2017 to promote the continuous development of national informatization [5]. With the development of artificial intelligence, the healthy life of artificial intelligence has become a new focus of social attention. In the new era of high-tech artificial intelligence, people's demand for aerobic and professional and technical talents is also increasing [6]. As the training base of professional aerobic talents, the ability level of aerobic professionals trained in colleges and universities not only affects the sustainable development of aerobics but also is related to the educational development of colleges and universities.

This paper analyzes and studies the application of the research on the talent training strategy of aerobic physical education under the background of artificial intelligence and holds that carrying out aerobic physical exercise can make people's life healthy, strong, and full of vitality and creativity, complement school physical education, comprehensively enhance college students' physique, and guide college students to pursue health and beauty. It has effectively resisted the erosion of negative decadent thoughts on campus culture. The arrival of aerobic physical education in the era of artificial intelligence also makes us realize that high-tech technology will have an increasing impact on the teaching ecology. In this paper, the visual capture of aerobic performance actions, through the selected data processing of aerobic actions, corrects the subtle differences of body movements in aerobic performance, specifies a standardized system for aerobic performance, learning, and adjudication, and paves the way for the development of aerobics.

The intelligent development of technology makes learning no longer passive acceptance, but a process of continuous information understanding and knowledge construction in a variety of learning experiences. Based on the application of intelligent sports, this paper discusses the application prospect of artificial intelligence technology in the talent training strategy of aerobic physical education.

The article "Research on the Training Strategy of Aerobic Physical Education Talents under the Background of Artificial Intelligence Era" was retracted in 2023. Reasons: signs of a paper mill; suspected computer-generated content; unreliable results or conclusions; lack of ethics approval or compliance.

## 2. Aerobic Evaluation System Based on Artificial Intelligence Gait Recognition

Under the background that national fitness and artificial intelligence have become national strategies, China's intelligent sports education platform has developed rapidly, and sports fitness has quietly entered the era of intelligent sports. As a new sports product, intelligent sports education products have developed rapidly, but there are many problems, such as single sports data collection method, lack of sports data mining, serious product homogenization, and insufficient product function development [7]. In order to better analyze the development status and problems of aerobic physical education talent training strategy research and application under the background of artificial intelligence era, the aerobic evaluation system of artificial intelligence gait recognition is analyzed as follows.

In Figure 1, the image information obtained by three cross-view cameras forms a three-dimensional dynamic real-time model through smart3d. The model extracts the skeleton frame information and action information through two columns of the extraction algorithm to form two array data and then outputs the evaluation results through the fuzzy neural network (FNN) module based on the sixth-order polynomial depth iterative regression algorithm. If using FNN to control the recent changes of timing data, or need to use the minimum node quantity data fuzzy convolution, the need to use the function curve is more complex and richer polynomial regression coefficient 6-order polynomial depth iterative regression basis function, based on sixth-order polynomial depth iterative regression FNN algorithm base function such as

(1) $$\begin{array}{c} y=\overset{n}{\underset{i=1}{\sum }}\overset{5}{\underset{j=0}{\sum }}A_{j}x_{i}^{j}, \end{array}$$

where *i* is the traversal pointer; *N* is the total number of nodes of the previous neural network; *x*_*i*_^*j*^ is the *j*th power of the input value of the *i*th node in the upper neural network; *y* is the output value of the neural network node; *A*_*j*_ is the coefficient to be regressed of the *j*th order polynomial, that is, each node in the formula contains 6 coefficients to be regressed from *A*_0_ to *A*_5_; *j* is the polynomial order.

The above extraction algorithm belongs to a relatively complex four-dimensional spatiotemporal array data extraction mode, that is, three rectangular spatial coordinate axes and one time axis data are convoluted in the *x*, *y*, and *z* axes, respectively, and then, a group of arrays is obtained by using the linear fuzzy algorithm. The above extraction algorithm transforms the four-dimensional spatiotemporal matrix into a one-dimensional directionless matrix at the statistical level, as shown in Figure 2.

The article "Research on the Training Strategy of Aerobic Physical Education Talents under the Background of Artificial Intelligence Era" was retracted in 2023. Reasons: signs of a paper mill; suspected computer-generated content; unreliable results or conclusions; lack of ethics approval or compliance.

Figure 2 shows the internal structure of skeleton frame module and action module in Figure 1. The folding algorithm is a log depth iterative regression neural network module, and the basis function is as shown in

(2) $$\begin{array}{c} y=\overset{n}{\underset{i=1}{\sum }}\left(A∙\log x_{i}+B\right), \end{array}$$

where *A* and *B* are coefficients to be regressed; the meanings of other mathematical symbols are the same as those above.

After the folding algorithm, it is necessary to enter the linear fuzzy module again for defuzzification. The linear fuzzy algorithm is to obtain the parallel difference matrix from the one-dimensional matrix and then cross calculate the two matrices to output a landmark result. The difference matrix calculation function is shown in

(3) $$\begin{array}{c} S\left\{t_{n\prime }\right\}⟶S\left\{\frac{t_{n}-t_{n-1}}{t_{n-1}}\right\},\;n^{\prime }\in \left\{0,1,2,3\cdots n\right\},n\in \left\{1,2,3\cdots n\right\}. \end{array}$$

The basis function of the linear fuzzy algorithm is shown in

(4) $$\begin{array}{c} F=S\left(t_{n}\right)∙S\left(\frac{t_{n}-t_{n-1}}{t_{n-1}}\right), \end{array}$$

where *S*{*t*_*n*′_} is the real-time value; *S*{(*t*_*n*_ − *t*_*n*−1_)/*t*_*n*−1_} indicates the difference ratio. The linear fuzzy matrix is input to the single-layer binarization, and the output result on a [0,1] interval is output: (0.9,1.0] red; (0.8,0.9] orange; (0.7,0.8] yellow; (0.6,0.7] blue; [0.0,0.6] no warning.

The three-dimensional spatial array processed by linear fuzzy module is used as the input data of subsequent FNN module, and the output data of FNN module is the objective evaluation result of artificial intelligence on aerobic performance. When students directly participate in the performance, the result is the performance score of students; when students participate in the referee, the system is used to provide the objective reference value of the players' performance results; when students participate in simulation teaching, the system is used to objectively evaluate the results of simulation students.

The result is the student's performance when the student is directly involved in the performance; the system is used to provide an objective reference value for the performance when the student participates and the objective evaluation of the performance when the student participates in simulation teaching.

## 3. Students Participating in Teaching Reform and Teaching Methods

### 3.1. Students

According to the method of average grouping, the students in the dance department of a college of physical education in Anhui are divided into two groups: the reference group using traditional education methods and the observation group using artificial intelligence teaching. 120 dance students enrolled from 2016 were randomly selected as the research objects of traditional teaching methods, including 92 girls and 28 boys, with an average age of 20.2 years; 120 dance students enrolled in 2017 were randomly selected as the analysis and research object of artificial intelligence teaching, including 87 girls and 33 boys, with an average age of 20.8 years.

The article "Research on the Training Strategy of Aerobic Physical Education Talents under the Background of Artificial Intelligence Era" was retracted in 2023. Reasons: signs of a paper mill; suspected computer-generated content; unreliable results or conclusions; lack of ethics approval or compliance.

### 3.2. Teaching and Assessment Methods

The research and analysis results of 2019 graduates using traditional teaching methods are that the traditional teaching methods and assessment methods are very single, fixed, and repeated, and students' understanding, learning habits, and interests are not conducive to stimulating and improving students' strong interest in practice.

The 2020 graduates adopt the teaching method based on the evaluation of artificial intelligence aerobics and conduct comprehensive evaluation by using the artificial intelligence teaching method, intelligent performance method, and judgment method. It is found that artificial intelligence aerobic teaching can better stimulate students' learning enthusiasm and more diversified courses. It is the supplement and development of new physical education and enhances students' physical values. In the performance course, the artificial intelligence (AI) system simulates the performance score of students; in the referee course, the AI system provides the objective value of the performance results of the contestants and students; in the teaching course, the AI system makes an objective evaluation value for simulating students' performance.

### 3.3. Statistical Methods

Although 2019 students did not participate in artificial intelligence teaching, their examination videos were archived in the school, so the artificial intelligence evaluation system was used to reevaluate the on-site data of 2019 students' examination as the reference group data.

The student scores in the simulated classroom of the teaching course are compared and analyzed by the methods of arithmetic mean and standard deviation rate, as shown in

(5) $$\begin{array}{c} \sigma =\frac{1}{n-1}\sqrt{\overset{n}{\underset{i=1}{\sum }}{\left(x_{i}-\mu \right)}^{2}}, \end{array}$$

(6) $$\begin{array}{c} \mu =\frac{1}{n}\overset{n}{\underset{i=1}{\sum }}x_{i}, \end{array}$$

where *σ* is the calculation result of standard deviation rate of input sequence; *n* is the number of elements of the input sequence *x*; *x*_*i*_ is the *x* input value of the input sequence *x*; *μ* is the arithmetic mean of the input sequence *x*.

The article "Research on the Training Strategy of Aerobic Physical Education Talents under the Background of Artificial Intelligence Era" was retracted in 2023. Reasons: signs of a paper mill; suspected computer-generated content; unreliable results or conclusions; lack of ethics approval or compliance.

The comparison method of the two groups of results is bivariate *t* check under SPSS, *t* ⋯ ⋯ as shown in

(7) $$\begin{array}{c} t=\frac{\mu_{1}-\mu_{2}}{\sqrt{\left(\left(n_{1}-1\right)\sigma_{1}^{2}+\left(n_{2}-1\right)\sigma_{2}^{2}\right)/\left(n_{1}+n_{2}-2\right)∙\left(\left(1/n_{1}\right)+\left(1/n_{2}\right)\right)}}\left(5\right), \end{array}$$

where *μ*_1_ and  *μ*_2_ are the arithmetic mean of the two compared series; *n*_1_ and *n*_2_ are the number of elements of the two compared sequences; *σ*_1_ and *σ*_2_ are the standard deviation rate of two compared series (see formula (6) for details); *t* is the bivariate *t* verification result.

## 4. Statistics of Teaching Achievements

### 4.1. Comparison Results of Students' Aerobic Performance

Aerobic is a brand-new sport, which integrates gymnastics, dance, music, and other performance items in the form of a group, giving people the image of a combination of health, beauty, and strength as a whole. After introducing students' physical education, students' physical fitness and physique can develop healthily. Artificial intelligence education system used in the process of aerobics learning decrease the difficulty of aerobics learning, let the learning action essentials, music rhythm, group cooperation requirements improved. Also let the aerobics overall coordination and body language in the process of performance more strength and beauty, let the students' physical and form benign more development.

Through the follow-up survey of students participating in aerobic learning on the education platform after employment, we get the one-year work data and the data of employers' satisfaction with their performance, as shown in Table 1.

In Table 1, the AI and artificial scores were subjected to bivariate *t*-calibration, *t* < 10.000, *P* < 0.001, with significant statistical differences. Bivariate *t* check for entry and first semester, *t* < 10.000, *P* < 0.01, with significant statistical differences. When employment, the employer satisfied the aerobic students, entry and second semester conducted bivariate *t* check, *t* < 10.000, *P* < 0.00, *P* < 0.01, with significant statistical differences. Their performance data in work and study fully explained that the students participating in the education platform will have higher employer satisfaction.

In order to more intuitively reflect the employer's satisfaction with the work of students participating in aerobic learning on the education platform in the above table, visualize the data in the table to get Figure 3.

In Figure 3, through a year's analysis of the work performance of students participating in aerobic learning on the education platform, it can be seen that with the correction of students' movements, rhythm, and strength by artificial intelligence, students can better master the essentials of aerobics, give better play to the overall coordination and beauty, and increase the public's love for aerobics.

The article "Research on the Training Strategy of Aerobic Physical Education Talents under the Background of Artificial Intelligence Era" was retracted in 2023. Reasons: signs of a paper mill; suspected computer-generated content; unreliable results or conclusions; lack of ethics approval or compliance.

### 4.2. Comparison Results of Student Aerobic Referee Scores

Although aerobic is a kind of sport, the integration of dance movements makes the body language more powerful and rhythmic. If only professionals judge the standardization of their actions with their naked eyes, there will be some limitations. After introducing artificial intelligence into students' teaching, students' body movements, music rhythm, and strength will be displayed at a glance under the artificial intelligence system. Some subtle movements will be captured and fed back to the interface for analysis, so as to standardize the aerobic movement process, so as to provide judgment basis for students' future work and study.

Through the follow-up survey of students participating in aerobic learning on the education platform after employment, we get the one-year work data and the satisfaction data of the employer on its ruling, as shown in Table 2.

In Table 2, a bivariate *t*-test with artificial intelligence and artificial scoring, *t* < 10.000, *P* < 0.01, with significant statistical difference. A bivariate *t*-test was carried out in both the induction and the first semester, *t* < 10.000, *P* < 0.01, with significant statistical difference. When the students first joined the employment, the employer was generally satisfied with the judgment of the students participating in aerobic learning on the education platform. A bivariate *t*-test was carried out in both the induction and the second semester, *t* < 10.000, *P* < 0.01, with significant statistical difference. Through more comprehensive and systematic standardized course standards, provide standard basis for aerobic performance adjudication, avoid adjudication disputes, and increase the satisfaction of employers with students participating in aerobic learning on the education platform.

In order to more intuitively reflect the employer's satisfaction with the ruling results of students participating in aerobic learning on the education platform in the above table, visualize the data in the table to get Figure 4.

In Figure 4, the students participating in the aerobic learning of the education platform have carried out standardized learning in the school, brought the aerobic standards to their daily work, and standardized and quantified their performance, learning, and adjudication, which has brought convenience to their daily work and been recognized by the employer.

The article "Research on the Training Strategy of Aerobic Physical Education Talents under the Background of Artificial Intelligence Era" was retracted in 2023. Reasons: signs of a paper mill; suspected computer-generated content; unreliable results or conclusions; lack of ethics approval or compliance.

### 4.3. Comparison Results of Students' Aerobic Teaching Results

All learning achievements need to prove the superiority of their value with achievements. Through the statistics and comparison of the teaching achievement data of students participating in aerobic learning on the education platform, it is obtained as shown in Table 3.

In Table 3, a bivariate *t*-test with artificial intelligence and artificial scoring, *t* < 10.000, *P* < 0.01, with significant statistical difference. A bivariate *t*-test was carried out in the first semester and the second semester, *t* < 10.000, *P* < 0.01, with significant statistical difference, indicating that there was no aerobic learning on the education platform, there was no standardized standard for aerobics, and the teaching level was uneven; the bivariate *t*-test was carried out in the first and second semester, *t* < 10.000, *P* < 0.01, with significant statistical difference. After participating in aerobic learning on the education platform, students' aerobic level was significantly improved.

In order to more intuitively reflect the employer's satisfaction with the teaching results of participating in aerobic learning on the education platform in the above table, visualize the data in the table to get Figure 5.

In Figure 5, through the analysis of the teaching results of students participating in aerobic learning on the education platform after work, it can be concluded that after systematic and standardized education, the overall aerobic exercise process is clearer, is more beautiful, has stronger strength and rhythm, and has more attention.

## 5. Discussion on the Achievements of Teaching Reform

Through the above research, it can be seen that the overall coordination of aerobics is very important, especially the team cooperation program, which has higher requirements for the unity and standardization of all personnel. At the same time, we should also take into account the ability of innovation, creation, expressiveness, and aesthetics, which is bound to bring some difficulty to the group's expressiveness. This requires the unification of aerobic standards and the standardization of performance, so as to create the effect of the combination of elegance, strength, and rhythm in stage performance.

Lai and Jiang, through the methods of literature and logical analysis, comb the research methods of three types of artificial intelligence based on data, logic, and knowledge on physical education since 2000 and demonstrate that artificial intelligence promotes the development of physical education and improves personalized education [8]. According to Ma and Ma, artificial intelligence plays an important role in physical education. This paper solves the problems encountered in physical education through accurate diagnosis, process monitoring, personalized service, and intelligent feedback of artificial intelligence. It also puts forward the development prospect of artificial intelligence in physical education [9].

The article "Research on the Training Strategy of Aerobic Physical Education Talents under the Background of Artificial Intelligence Era" was retracted in 2023. Reasons: signs of a paper mill; suspected computer-generated content; unreliable results or conclusions; lack of ethics approval or compliance.

Through the introduction of artificial intelligence, the correction of body coordination of aerobic should be handled in detail, the actions of individuals in the group should be decomposed and returned one by one, the problems should be found, and the scoring of aerobic judges should be standardized and quantified, so as to make aerobics a standardized teaching, so as to have a ruler to weigh its standard in the learning, performance, and teaching of aerobics, paving the way for its development.

According to Yang, physical education is to improve students' physical quality, and it is also a stage for students to develop good exercise habits and high-quality physical fitness. With the emergence of big data and artificial intelligence, this paper discusses its application in intellectual education through the combination of intelligent sports and big data technology and puts forward the practical process of building a platform and application through artificial intelligence, giving each student personalized guidance and promotion, so as to improve the overall quality of the whole people [10].

Through the comparison between traditional teaching and artificial intelligence teaching, artificial intelligence teaching is obviously better than the previous traditional education system in daily performance, judgment, and teaching performance, provides a new cognitive aspect for students to learn aerobics in the future, specifies a standardized system for aerobic performance, learning, and judgment, and paves the way for the development of aerobics.

## 6. Summary

This paper compares the performance, judgment, and teaching performance of students participating in aerobic learning on the education platform; the traditional teaching methods and assessment methods are very single, fixed, and repeated. Students' understanding, learning habits, and interests are not conducive to stimulate and improve students' strong interest in practice. Using artificial intelligence teaching method, intelligent performance method, and referee method for comprehensive evaluation, artificial intelligence aerobic teaching can stimulate students' learning enthusiasm, and the curriculum is more diversified. It is the supplement and development of new physical education and enhances students' physical values. Therefore, obtaining the analysis data shows that the popularization of the education platform is obviously better than the previous traditional education system in daily performance, judgment, and teaching performance. It will provide a new cognitive aspect for students to learn aerobics in the future, and the follow-up research will also provide the evaluation effect of artificial intelligence on aerobics.

The article "Research on the Training Strategy of Aerobic Physical Education Talents under the Background of Artificial Intelligence Era" was retracted in 2023. Reasons: signs of a paper mill; suspected computer-generated content; unreliable results or conclusions; lack of ethics approval or compliance.

## Figures and Tables

**Figure 1:** Overall algorithm architecture.

**Figure 2:** Schematic diagram of extraction algorithm architecture.

**Figure 3:** Comparison chart of students' aerobic performance and employers' opinions.

**Figure 4:** Comparison of student aerobic referee scores and opinions of employers.

**Figure 5:** Comparison of students' aerobic teaching results and employers' opinions.

**Table 1:** Statistics of students' aerobic performance (the data comes from the student files of the student office of our university).

Grouping	Artificial intelligence	Manual scoring	Opinions of the employer		
			Induction	First semester	Second semester
2019	7.93 ± 0.85	8.32 ± 0.797	7.85 ± 0.76	8.23 ± 0.78	8.39 ± 0.81
2020	7.36 ± 0.78	8.39 ± 0.87	8.56 ± 0.83	9.14 ± 0.89	9.56 ± 0.87
*t*	4.85	66.14	5.23	5.78	6.18
*P*	0.006	0.013	0.005	0.006	0.007

Artificial intelligence: the crystallization of human wisdom through computer program technology; manual scoring: professionals judge the score with naked eyes through professional knowledge; entry: after being approved by the employing unit, the job seeker can enter the employing unit to start the probation process after being notified by the recruiting unit; first semester: the first semester after the beginning of school; second semester: the second semester after the beginning of school; *t*, *P* comes from the bivariate *t* check.

**Table 2:** Statistics of student aerobic referee scores (the data comes from the student files of the student office of our university).

Grouping	Artificial intelligence	Manual scoring	Opinions of the employer		
			Induction	First semester	Second semester
2019	7.79 ± 0.81	8.16 ± 0.75	7.95 ± 0.87	8.33 ± 0.74	8.67 ± 0.91
2020	7.23 ± 0.67	8.21 ± 0.85	8.48 ± 0.76	9.14 ± 0.89	9.43 ± 0.84
*t*	5.26	59.78	6.01	5.93	6.34
*P*	0.007	0.015	0.005	0.006	0.008

Artificial intelligence: the crystallization of human wisdom through computer program technology; manual scoring: professionals judge the score with naked eyes through professional knowledge; entry: after being approved by the employing unit, the job seeker can enter the employing unit to start the probation process after being notified by the recruiting unit; first semester: the first semester after the beginning of school; second semester: the second semester after the beginning of school; *t*, *P* comes from the bivariate *t* check.

The article "Research on the Training Strategy of Aerobic Physical Education Talents under the Background of Artificial Intelligence Era" was retracted in 2023. Reasons: signs of a paper mill; suspected computer-generated content; unreliable results or conclusions; lack of ethics approval or compliance.

**Table 3:** Statistics of students' aerobic teaching scores (the data comes from the student files of the student office of our university).

Grouping	Artificial intelligence	Manual scoring	Opinions of the employer		
			Induction	First semester	Second semester
2019	7.69 ± 065	8.23 ± 0.57	7.88 ± 0.82	8.45 ± 0.76	8.69 ± 0.79
2020	7.01 ± 0.74	8.35 ± 0.82	8.62 ± 0.92	9.19 ± 0.87	9.58 ± 0.93
*t*	4.86	62.17	5.24	6.03	6.42
*P*	0.006	0.017	0.007	0.008	0.007

Artificial intelligence: the crystallization of human wisdom through computer program technology; manual scoring: professionals judge the score with naked eyes through professional knowledge; entry: after being approved by the employing unit, the job seeker can enter the employing unit to start the probation process after being notified by the recruiting unit; first semester: the first semester after the beginning of school; second semester: the second semester after the beginning of school; *t*, *P* comes from the bivariate *t* check.

## Data Availability

The data underlying the results presented in the study are available within the manuscript.
